The article "Evidence-Based Care Can Improve Treatment Compliance and Quality of Life of Patients with Acute Pancreatitis" was retracted in 2023. Reason: concerns about the peer review.

# Evidence-Based Care Can Improve Treatment Compliance and Quality of Life of Patients with Acute Pancreatitis

**DOI:** 10.1155/2022/7621658

**Published:** 2022-02-12

**Authors:** Qiu Zheng, Li Cao, Huanhuan Ma, Yangyang Jin, Yufei Gao, Jiating Nie, Qingfeng Guo

**Affiliations:** ^1^Department of Gastroenterology, The Fourth Hospital of Harbin Medical University, Harbin 150001, Heilongjiang, China; ^2^Department of Cerebral Surgery, The Fourth Hospital of Harbin Medical University, Harbin 150001, Heilongjiang, China; ^3^Medical Oncology, The Fourth Hospital of Harbin Medical University, Harbin 150001, Heilongjiang, China; ^4^Heilongjiang University of Traditional Chinese Medicine, Harbin 150040, Heilongjiang, China; ^5^The Fourth Hospital of Harbin Medical University, Harbin 150001, Heilongjiang, China; ^6^Department of Nursing Care, The Fourth Hospital of Harbin Medical University, Harbin 150001, Heilongjiang, China

## Abstract

Acute pancreatitis represents a disease characterized by acute necro-inflammatory changes in the pancreas, which is histologically characterized by destruction of alveolar cells. We aim to explore whether evidence-based care can improve treatment compliance and quality of life of patients with acute pancreatitis. The changes of hemoglobin (HGB), serum pre-albumin (PAB), and serum albumin (ALB) before and after care were observed, as well as the incidence of complications after care, total effective rate after care, disease severity (bedside index for severity in acute pancreatitis, BISAP) before and after care, and psychological scores of the two groups before and after care were observed. Patients' compliance after care, self-management scores after care, and quality of life after care were compared between the two groups. After care, HGB, PAB, and ALB increased significantly in both groups (*p* < 0.05) and were higher in OG than CG. Compared with CG, OG had significantly lower incidence of complications (*p*=0.009), significantly higher total effective rate (*p*=0.011), significantly lower disease severity (*p* < 0.05), significantly better psychological condition scores (*p* < 0.05), significantly higher compliance scores (*p* < 0.05), higher self-management scores (*p* < 0.05), and significantly higher quality of life (*p* < 0.001). Evidence-based care can improve treatment compliance of patients with acute pancreatitis and can effectively improve their quality of life.

## 1. Introduction

Acute pancreatitis is a common digestive system disease, which is caused by abnormal digestive enzymes in the patient's own organs, resulting in inflammation of the pancreatic secretions [1]. The age range of the disease is wide, but most of the people who develop it are adults [2]. According to data, the incidence of acute pancreatitis is 34 cases per 100,000 in the general population and is increasing worldwide, and its incidence increases with age [3]. The main symptoms of acute pancreatitis are sudden onset of upper abdominal pain accompanied by nausea and vomiting [4], while patients with severe acute pancreatitis may be accompanied by hypotension or shock, leading to organ dysfunction and high mortality [5]. Patients need to be hospitalized immediately for diagnosis and treatment of the disease. Usually, symptomatic treatment and nonsurgical treatment are the main treatment methods [6]. Although most patients with acute pancreatitis have mild conditions and better treatment methods, there are still some patients with severe acute pancreatitis and the complications after treatment are very difficult [7]. Surgical treatment is required for complications, and the prognosis is poor [8]. Clinical data show that severe pancreatitis has a rapid onset and the patient is in dangerous condition, which causes a serious burden on pancreas, reduces patients' quality of life, and even endangers life [9].

The article "Evidence-Based Care Can Improve Treatment Compliance and Quality of Life of Patients with Acute Pancreatitis" was retracted in 2023. Reason: concerns about the peer review.

Chronic alcohol ingestion, cholelithiasis, and overeating are usually the main causes of acute pancreatitis [10]. Therefore, choosing an appropriate nursing method is particularly important to improve the rehabilitation of acute pancreatitis and to avoid the continuous deterioration of the disease [11]. Over the past decade, cares in China have continued to shine in the treatment of clinical diseases, improving poor patient outcomes and enhancing the relationship between doctors and nurses [12], which greatly improves treatment compliance of patients and enhances treatment effects [13]. A review of previous studies suggested that evidence-based care based on evidence-based medicine is effective in constraining patient self-management and reducing disease complications [14]. Acute pancreatitis represents a disease characterized by acute necro-inflammatory changes in the pancreas, which is histologically characterized by destruction of alveolar cells [15]. It is found that acute pancreatitis secondary to alcohol is more common in men and gallstone pancreatitis is more common in women [16]. At present, mild acute pancreatitis is usually treated with drugs, and the prognosis is generally good [17]. Moderate and severe acute pancreatitis should be treated according to the cause of disease, and if necessary, surgery should be performed, and the prognosis is generally poor due to frequent complications [18].

Besides, there are few clinical studies on the intervention effect of evidence-based care on patients with acute pancreatitis. Therefore, this experiment analyzes the effect of evidence-based care on patients with acute pancreatitis and observes the improvement of patients' compliance and quality of life, aiming at providing effective care for future clinical diagnosis and treatment of acute pancreatitis, so as to increase its recovery rate.

The article "Evidence-Based Care Can Improve Treatment Compliance and Quality of Life of Patients with Acute Pancreatitis" was retracted in 2023. Reason: concerns about the peer review.

## 2. Materials and Methods

With deeper cognition of diseases and master of previous experience, the nursing staff can realize the adverse reactions of patients in time, adjust treatment strategies, closely cooperate with doctors, and improve the treatment effects from the patient's point of view [19], which is also suspected to be the main reason for the obvious improvement of disease status in OG after implementing care. Author Aviles et al. [20] pointed out that evidence-based care is of great help to promote the recovery of diseases by analyzing the effects of evidence-based care on enhancing the recovery of patients undergoing duodenectomy, which is similar to our experimental results.

A total of 117 patients with severe acute pancreatitis treated in our hospital from May 2017 to June 2019 were collected for prospectively analyzed, 65 of whom receiving evidence-based care during treatment were enrolled in the observation group (OG), and the other 52 patients receiving routine care during treatment were enrolled in the control group (CG). Note: this study has been approved by the Ethics Committee of our hospital.

### 2.1. Inclusion and Exclusion Criteria

Inclusion criteria were as follows: patients were diagnosed as severe acute pancreatitis after laboratory and imaging examination according to Chinese Journal of Pancreatology, patients were over 25 years old, patients underwent operation in our hospital, with stable vital signs, complete clinical data, and were in rehabilitation stage, and patients and their families knew and agreed to this experiment.

Exclusion criteria were as follows: patients had abnormal liver or renal function, other congenital diseases, or major diseases, patients did not have the ability to read and write, patients had immune dysfunction, and patients had drug allergy.

### 2.2. Nursing Methods

The team of Williams [21] also proposed that evidence-based care can effectively improve the recovery of patients after cardiac surgery, which has application value and supports this study. CG: routine care was adopted. The patients were assigned to the ward when they were admitted to the hospital. Then, the nursing staff followed the doctor's advice to monitor the vital signs of patients, performed routine examinations, made preparations before operation, and explained simple disease knowledge to the patients and their families. Besides, the nursing staff reminded patients of matters needing attention, performed routine care operations after operation, dispensed drugs, paid attention to the progress of the disease, and guided and restrained the behaviors and habits of the patients such as diet after operation.

The article "Evidence-Based Care Can Improve Treatment Compliance and Quality of Life of Patients with Acute Pancreatitis" was retracted in 2023. Reason: concerns about the peer review.

OG: evidence-based care was given on the basis of routine care in CG. The nursing staff paid close attention to the patient's heart rate, blood pressure, and other vital signs before surgery, actively cooperated with the attending physician, registered, and completed the preoperative examination. The nursing staff should search for evidence based on previous nursing experience of acute pancreatitis and relevant literature, deepen their understanding of diseases, set reasonable care measures according to patients' own conditions, carry out disease education, psychological decompression, restrain misconduct, and perform other interventions, and closely grasp patients' first-hand information during and after operation. According to the patient's own situation and the requirements of the corresponding attending physician, the patient was given medication and diet control. The recovery of patients was also closely monitored by the nursing staff.

### 2.3. Outcome Measures

In the implementation of evidence-based care, nursing staff should closely observe patients' emotional changes, tell successful cases to patients before operation, enhance patients' self-confidence, reasonably regulate patients' diet and living habits after operation, and increase the doctor-patient relationship, so as to improve patients' cooperation and promote the treatment process [22]; the above are important factors in the value of evidence-based care. The changes of hemoglobin (HGB), serum pre-albumin (PAB), and serum albumin (ALB) before and after care were observed, as well as the incidence of complications after care, total effective rate after care, disease severity (bedside index for severity in acute pancreatitis, BISAPe) [23] before and after care, and psychological scores of the two groups before and after care were observed. Patients' compliance after care, self-management scores [24] after care, and quality of life after care were compared between the two groups.

### 2.4. Statistical Methods

All statistical analysis of the experimental results was performed by using SPSS24.0 statistical software (Shanghai Yuchuang Network Technology Co., Ltd.). All graph results were plotted by Graphpad8 (SOFTHEAD Inc., Shenzhen). Enumeration data were expressed in the form of (%), and chi-square test was utilized for intergroup comparison. Measurement data were expressed in the form of (mean ± standard deviation), and *t*-test was used for intergroup comparison. Univariate analysis of variance (ANOVA) and LSD back testing were used for comparison among multiple groups. Repeated measures ANOVA and Bonferroni back testing were used for comparison between multiple time points. *p* < 0.05 was considered statistically significant.

The article "Evidence-Based Care Can Improve Treatment Compliance and Quality of Life of Patients with Acute Pancreatitis" was retracted in 2023. Reason: concerns about the peer review.

## 3. Results

### 3.1. Patient Data

There was no statistic difference in age, gender, BMI, living environment, eating habits, smoking history, drinking history, family medical history, ethnicity, C-reactive protein, white blood cells, and so on (*p* > 0.05) as shown in Table 1.

### 3.2. Changes of HGB, PAB, and ALB in Two Groups before and after Care

The changes of HGB, PAB, and ALB before and after care were detected. The results showed that there was no statistic difference between the two groups before care (*p* > 0.05), but after care, HGB, PAB, and ALB in both groups increased (*p* < 0.05) and were higher in OG than CG (*p* < 0.05) as shown in Figure 1.

### 3.3. Incidence of Complications in Two Groups after Care

The incidence of complications after care in the two groups was observed. The total incidence of adverse reactions in OG was 2 (3.08%), while that in CG was 9 (17.31%), which was significantly lower in OG than CG (*p*=0.009) as shown in Table 2.

### 3.4. Effective Rate of the Two Groups after Care

The effective rates of the two groups were observed after care. The markedly effective rate of OG was 75.38%, effective rate was 23.08%, and ineffective rate was 1.54%, with a total effective rate of 98.46%. The markedly effective rate of CG was 42.31%, effective rate was 44.23%, and ineffective rate was 13.46%, with a total effective rate of 86.54%. The total effective rate of OG was significantly higher than that of CG (*p*=0.011) with statistic difference as shown in Table 3.

### 3.5. The Severity of Diseases in the Two Groups before and after Care

BISAP was used to analyze the disease severity before and after care. The results showed that there was no remarkable difference between the two groups before care (*p* > 0.05), but the scores of both groups decreased after care and were notably lower in OG than CG (*p* < 0.05) as shown in Figure 2.

### 3.6. Psychological Scores of the Two Groups before and after Care

The psychological status of the two groups of patients before and after care was observed. The results showed that there was no remarkable difference in psychological scores between the two groups before care (*p* > 0.05), but the psychological status scores of the two groups decreased after care, which were lower in OG than in CG (*p* < 0.05) as shown in Figure 3.

The article "Evidence-Based Care Can Improve Treatment Compliance and Quality of Life of Patients with Acute Pancreatitis" was retracted in 2023. Reason: concerns about the peer review.

### 3.7. Comparison of Patients' Compliance after Care between the Two Groups

Comparison of the patients' compliance after care between the two groups showed that the compliance score of OG was notably higher than that of CG (*p* < 0.05) as shown in Figure 4.

### 3.8. Comparison of Self-Management Scores between the Two Groups after Care

After care, the self-management scores of patients in the two groups were observed. The results showed that the scores of disease management, diet management, medication management, and rehabilitation exercise management in OG were higher than those in CG, with statistical difference (*p* < 0.05) as shown in Figure 5.

### 3.9. Changes of Quality of Life after Care in Two Groups

By observing the quality of life of the two groups of patients after care, it could be seen that the scores of physical function, role physical, emotional function, cognitive function, social function, and other dimensions of the quality of life of the observation group after care were significantly higher than those of the control group (*p* < 0.05) as shown in Table 4.

## 4. Discussion

According to statistics, the mortality rate of patients with acute pancreatitis is estimated to be 5% [6], which seriously threatens the patient's life safety. It is known that poor diet and lifestyle are important factors in the onset of acute pancreatitis, so it is extremely important to improve bad habits after treatment for patients' rehabilitation, and a large number of documents have proved that effective care can effectively improve patients' quality of life during disease recovery period [25]. Therefore, this study focuses on evidence-based care in acute pancreatitis to improve patients' treatment compliance and quality of life, and the results are as follows: firstly, the changes of HGB, PAB, and ALB before and after care were detected. The results showed that there was no statistical difference between the two groups before care, but after care, HGB, PAB, and ALB in both groups increased and were higher in OG than CG, suggesting that evidence-based care can obviously improve the serum indexes of patients and promote the curative effect. We speculate that its value lies in the fact that evidence-based care follows the basis of evidence-based medicine, and patients can be treated according to different situations, including nutritional agent adjustment according to individual physical abnormalities and rational nutrition supply, so as to improve serum indexes and promote curative effects.

The incidence of complications after care in the two groups was observed. The total incidence of adverse reactions in OG was 2 (3.08%), while that in CG was 9 (17.31%), which was significantly lower in OG than CG (*p*=0.009). The results indicated that evidence-based care can effectively improve prognosis of patients and reduce complications. Comparison of effective rate showed that the total effective rate of OG was 98.46%, which was notably higher than that of CG (86.54%), showing that evidence-based care has high clinical nursing value. We speculate that it is the efficient evidence finding of evidence-based care, summarizing previous care experiences, refining previous deficiencies, and formulating reasonable nursing interventions based on the individual's physical condition, thus further reduced the risk of complications and achieved consolidation of treatment outcomes. Then, we applied BISAP to analyze the degree of disease recovery before and after care. The results showed that there was no remarkable difference in BISAP between the two groups before care, but after care, the scores of both groups were reduced and were significantly lower in OG than CG, suggesting that evidence-based care can significantly reduce the severity of disease and relieve the pain of patients. Evidence-based care refers to the intervention of patients by consulting relevant disease data and combining with the actual situation of patients. Observation of psychological status of the two groups of patients before and after care showed that there was no remarkable difference in psychological scores between the two groups before care, but the psychological status scores of the two groups decreased after care, which were lower in OG than in CG. This result exemplifies the importance of evidence-based care in relieving patients' stress, anxiety, and other negative emotions. Comparison of the patients' compliance after care between the two groups also showed that the compliance score of OG was notably higher than that of CG, better reflecting the people-centered, comprehensive, and holistic interventions of evidence-based care. Finally, we observed the scores of self-management and the quality of life of patients in the two groups after care. The results showed that the scores of disease management, diet management, medication management, and rehabilitation exercise management in OG were higher than those in CG, and the quality of life was obviously better in OG than CG which further confirmed our above conjecture and showed that evidence-based care greatly improved the treatment outcome of patients.

The article "Evidence-Based Care Can Improve Treatment Compliance and Quality of Life of Patients with Acute Pancreatitis" was retracted in 2023. Reason: concerns about the peer review.

## 5. Conclusion

In conclusion, evidence-based care can improve treatment compliance of patients with acute pancreatitis and can effectively improve their quality of life.

However, there are still some shortcomings in this experiment. For example, there are many nursing methods in clinic; the best nursing mode is still controversial. And the research objects in this paper are severe pancreatitis patients; it is not excluded that the application of evidence-based care in other diseases may be different from the experimental results. In addition, the time of this study was short, and long-term follow-up was not conducted. Hence, we will expand the sample size of the study as soon as possible, extend the experimental period, and conduct more detailed and comprehensive experimental analysis to obtain more perfect experimental results.

## Figures and Tables

**Figure 1:** Changes of HGB, PAB, and ALB before and after care between observation group and control group. (a) HGB changes before and after care. (b) PAB changes before and after care. (c) ALB changes before and after care. *Note.*^*∗*^denotes comparison with before care; & denotes comparison with observation group.

**Figure 2:** Recovery degree of the two groups before and after care. *Note.*^*∗*^denotes comparison with before care; & denotes comparison with observation group.

**Figure 3:** Psychological scores of two groups before and after care. (a) SAS score of the two groups before and after care. (b) SDS score of the two groups before and after care. *Note*. ^*∗*^denotes comparison with before care; & denotes comparison with observation group.

**Figure 4:** Comparison of patients' compliance after care between the two groups.

**Figure 5:** Comparison of self-management scores between two groups after care. (a) The score of disease management in the two groups after care. (b) The score of diet management in the two groups after care. (c) The score of medication management in the two groups after care. (d) The score of rehabilitation exercise management in the two groups after care.

**Table 1:** General data between observation group and control group (*n* [%]).

	Observation group (*n* = 65)	Control group (*n* = 52)	*t* or *x*^2^	*p*
Age (years)			0.246	0.806
	46.8 ± 8.6	47.2 ± 8.9		
Gender			0.267	0.605
Male	43 (66.15)	32 (61.54)		
Female	22 (33.85)	20 (38.46)		
BMI (kg/cm^2^)			0.748	0.456
	25.62 ± 3.05	26.16 ± 4.72		
Living environment			0.067	0.796
Town	41 (63.08)	34 (65.38)		
Countryside	24 (36.92)	18 (34.62)		
Dietary habit			0.007	0.933
Good	28 (43.08)	22 (42.31)		
Poor	37 (56.92)	30 (57.69)		
Smoking history			0.032	0.859
Present	44 (67.69)	36 (69.23)		
Absent	21 (32.31)	16 (30.77)		
Drinking history			0.178	0.673
Present	40 (61.54)	30 (57.69)		
Absent	25 (38.46)	22 (42.31)		
Family medical history			0.086	0.769
Present	10 (15.38)	7 (13.46)		
Absent	55 (84.62)	45 (86.54)		
Ethnicity			0.491	0.484
Han	56 (86.15)	47 (90.38)		
Minority	9 (13.85)	5 (9.62)		
C-reactive protein (mh/L)			0.142	0.888
	23.12 ± 5.34	23.26 ± 5.29		
White blood cell (×10^9^/L)			1.121	0.265
	14.64 ± 2.31	15.11 ± 2.18		

The article "Evidence-Based Care Can Improve Treatment Compliance and Quality of Life of Patients with Acute Pancreatitis" was retracted in 2023. Reason: concerns about the peer review.

**Table 2:** Adverse reaction rate after care between observation group and control group [*n* (%)].

	Observation group (*n* = 65)	Control group (*n* = 52)	*x* ^2^	*p*
Respiratory disorder				
	0 (0.00)	1 (1.92)		
Impaired cardiac function				
	0 (0.00)	2 (3.85)		
Gastrointestinal hemorrhage				
	1 (1.54)	3 (5.77)		
Renal dysfunction				
	1 (1.54)	3 (5.77)		
Total (%)			6.868	0.009
	2 (3.08)	9 (17.31)		

**Table 3:** Total effective rate of the two groups after care between observation group and control group [*n* (%)].

	Observation group (*n* = 65)	Control group (*n* = 52)	*x* ^2^	*p*
Markedly effective				
	49 (75.38)	22 (42.31)		
Effective				
	15 (23.08)	23 (44.23)		
Ineffective				
	1 (1.54)	7 (13.46)		
Total effective rate			6.447	0.011
	64 (98.46)	45 (86.54)		

**Table 4:** Comparison of quality of life between the two groups.

	Observation group (*n* = 65)	Control group (*n* = 52)	*t* value	*p* value
Physical function			13.010	<0.001
	91.23 ± 3.26	83.22 ± 3.37		
Role physical			21.020	<0.001
	85.52 ± 3.56	72.30 ± 3.14		
Emotional function			25.510	<0.001
	86.53 ± 3.25	70.74 ± 3.42		
Cognitive function			12.690	<0.001
	91.43 ± 3.59	83.34 ± 3.21		
Social function			21.640	<0.001
	65.55 ± 3.18	52.64 ± 3.24		

## Data Availability

The datasets used and/or analyzed during the current study are available from the corresponding author on reasonable request.
